RETRACTED

# Changes of Entropy Index and Cerebral Oxygen Metabolism in the Maintenance of Remifentanil Anesthesia and Their Predictive Value for Postoperative Hyperalgesia

**DOI:** 10.1155/2022/1080858

**Published:** 2022-03-11

**Authors:** Tianhao Zhang, Fang Ma

**Affiliations:** ^1^Department of Anesthesiology, The 1st Hospital of China Medical University, Shenyang, Liaoning 110000, China; ^2^Cancer Hospital of China Medical University, Liaoning Cancer Hospital & Institute, Shenyang, Liaoning 110801, China

## Abstract

**Objective:**

To explore the changes of entropy index and cerebral oxygen metabolism in the maintenance of remifentanil anesthesia and the predictive value of postoperative hyperalgesia.

**Methods:**

A total of 266 patients undergoing general anesthesia in our hospital from January 2020 to October 2021 were selected, and remifentanil was used to maintain anesthesia. The state entropy, reaction entropy, and cerebral oxygen metabolism indexes (cerebral oxygen uptake rate (CERO_2_), arterial-venous blood oxygen difference (Da-jvO_2_)) of patients before induction of anesthesia, 15 minutes during the operation, and at the end of the operation were compared. The influencing factors of postoperative hyperalgesia were analyzed. The logistic regression model of postoperative hyperalgesia was established, and the value of entropy index and cerebral oxygen metabolism in predicting postoperative hyperalgesia was evaluated by drawing the receiver operating characteristic curve (ROC).

**Results:**

The state entropy, response entropy, and CERO_2_ at 30 min during the operation and at the end of the operation were lower than those before the induction of anesthesia, and Da-jvO_2_ was higher than that before the induction of anesthesia (*P* < 0.001). At the end of the operation, the state entropy, reaction entropy, and CERO_2_ were higher than 30 minutes during the operation, and Da-jvO_2_ was lower than 30 minutes during the operation (*P* < 0.001). The dosage of remifentanil, reaction entropy, and CERO_2_ at the end of the operation entered the logistic model. The AUC value of the reaction entropy and CERO_2_ combined to predict postoperative hyperalgesia at the end of the operation was 0.851 greater than the reaction entropy at the end of the operation (*χ*^2^ = 3.847, *P* = 0.036), CERO_2_ (*χ*^2^ = 2.589, *P* = 0.010) single index predictive value.

**Conclusion:**

The entropy index and cerebral oxygen metabolism in general anesthesia patients change with the progress and discontinuation of remifentanil maintenance anesthesia, and the combination of the two has a high predictive power in postoperative hyperalgesia risk assessment. When the reaction entropy > 54.23, CERO_2_ > 34.14%, or the total dosage of remifentanil ≥ 30 *μ*g/kg at the end of the operation, we should be highly vigilant of the occurrence of postoperative hyperalgesia and postoperative analgesia management should be strengthened.

RETRACTED

## 1. Introduction

Remifentanil is a *μ*-opioid receptor agonist, which has the characteristics of rapid onset, short half-life, remarkable analgesic effect, and high safety. Remifentanil does not depend on liver and kidney metabolism and will not accumulate in the body after long-term infusion, so it is widely used in surgical anesthesia, whether it is daytime surgery or complicated large-scale surgery [1–3]. However, the analgesic effect of remifentanil disappears rapidly after stopping the drug, which will induce hyperalgesia, lead to severe discomfort after the operation, increase the dosage of analgesic drugs, delay the postoperative recovery, and prolong the hospital stay [4]. At present, there is a lack of standardized diagnostic criteria and preventive measures for remifentanil-induced hyperalgesia in clinic, which brings great challenges to postoperative pain management. Although there have been cohort studies on postoperative hyperalgesia caused by remifentanil, it is not known whether the risk of postoperative hyperalgesia can be predicted by specific indicators due to individual heterogeneity [5]. Entropy index can accurately reflect the anesthesia depth of surgical patients with high sensitivity and can avoid the influence of posture change [6]. The indexes of cerebral oxygen metabolism are mainly used to judge the oxygen consumption status of patients' brain tissue, and the relationship between cerebral hypoxia and pain response has been reported [7]. Based on this, this study detects the entropy index and cerebral oxygen metabolism index of anesthesia patients maintained by remifentanil and analyzes its value in predicting postoperative hyperalgesia, aiming at providing guidance for pain management of patients undergoing surgery. The specific results are reported as follows.

## 2. Materials and Methods

### 2.1. Object of Study

A total of 266 patients undergoing general anesthesia in our hospital from January 2020 to October 2021 were selected. Remifentanil was used to maintain anesthesia. Inclusion criteria are as follows: (1) all patients were under general anesthesia; (2) American Association of Anesthesiologists (ASA) grade i~iii; (3) the estimated operation time is more than >30 min; and (4) patients or family members know about this study and sign the consent form. Exclusion criteria are as follows: (1) preoperative mental disorder, (2) history of drug dependence, (3) cardiovascular and cerebrovascular diseases or nervous system diseases, (4) high airway reactivity, (5) history of epilepsy, (6) abnormal EEG and EMG before operation, and (7) taking antidepressant and sedative drugs before operation. This study was approved by the hospital ethics committee.

RETRACTED

### 2.2. Methods

(1) After entering the room, clean the forehead, remove the grease, connect the entropy index monitor connection module (GE Healthcare Finland Oy company; M-Entropy, S/5tm; Datex Ohmeda; Finland), place the electrode in the middle of the forehead, and record the state entropy and reaction entropy before anesthesia induction, 30 min during operation and at the end of operation. (2) Before induction of anesthesia, 30 minutes during the operation, and at the end of the operation, 1 ml each of the patient's internal jugular venous bulb and internal carotid radial artery blood were collected. Blood Gas Biochemical Analyzer (Beijing Perlong New Technology Co., Ltd., PL2000PLUS, China) was used to measure the blood oxygen saturation (SjvO2) of the internal jugular venous bulb (PjvO2), arterial blood oxygen saturation (SaO2), and the partial pressure of arterial blood oxygen (PaO2). An automatic hematology analyzer (Mindray Medical International Co., Ltd., BC-5000, China) was used to determine the level of hemoglobin (Hb). Internal carotid artery blood oxygen content (CaO2) = 1.36 × Hb × SaO2 + PaO2 × 0.0031, internal jugular vein blood oxygen content (cjvo2) = 1.36 × Hb × SjvO2 + +PjvO2 × 0.0031, arterial venous oxygen content difference (Da − jvO_2_) = CaO2 − cjvo2, and cerebral oxygen uptake rate (CERO_2_) = (SaO2 − SjvO2)/SaO2 × 100%.

### 2.3. Observation Index

(1) State entropy, reaction entropy, CERO_2_, and Da-jvO_2_ were compared before anesthesia induction, 15 min during operation, and at the end of operation. (2) Statistic the postoperative hyperalgesia of patients, and compare the incidence of postoperative hyperalgesia of different patients. The following two items are judged as hyperalgesia [8]. (a) After entering the anesthesia recovery room for 15 min and 45 min, the pain area of the wound is measured by acupuncture, and the pain area at 45 min is 1 cm larger than that at 15 min (if there are multiple wounds, the largest wound is the test point). (b) Sustained severe pain occurred locally in the wound, which was assessed by visual analogue scale (VAS) to be over 8 points, but was ineffective after placebo treatment. Fentanyl 1 *μ*g/kg was injected intravenously before leaving the anesthesia recovery room. (c) Wipe gently with dry cotton ball and alcohol cotton ball in the pain area (avoiding the wound), and the VAS score increases by ≥2 points. (d) The degree of pain is not consistent with clinical severity. (e) Limb protective action. (f) The VAS score again at 4 h and 24 h after operation was >8. (g) Any other time needs to be handled by anesthesiologists. (3) Analyze the influencing factors of postoperative hyperalgesia. (4) The logistic regression model of postoperative hyperalgesia was established and evaluated. (5) Evaluate the value of entropy index and cerebral oxygen metabolism in predicting postoperative hyperalgesia.

RETRACTED

### 2.4. Statistical Treatment

SPSS (25.0 for Windows) statistical software was used to analyze the data. Kolmogorov-Smirnov normality test of measured data accords with normal distribution, described by ($\bar{x}\pm s$). Paired *t*-test is used for comparison of different time indexes, the number of cases (percentage) is used for counting data, and *χ*^2^ test is used for both sides' test, with *α* = 0.05 as the test level. The factors with *P* < 0.05 in univariate analysis are tested for multicollinearity. When the variance inflation factor (Vif) is less than 5, it is considered that there is no multicollinearity. Logistic multivariate correlation analysis and Hosmer-Lemeshow test model fit degree are included. The receiver operating characteristic curve (ROC) drawn by MedCalc 11.4 was used to analyze the predictive value of entropy index and cerebral oxygen metabolism index on postoperative hyperalgesia, and the area under the curve (AUC) was obtained. Logistic binary regression fitting was used for joint prediction, and the predictive probability logit (*P*) was returned as an independent test variable. The AUC differences of different indexes were compared by Delong nonparametric method, with *α* = 0.05 as the inspection level.

## 3. Result

### 3.1. Comparison of Entropy Index and Cerebral Oxygen Metabolism before and after Anesthesia

The state entropy, reaction entropy, and CERO_2_ at the end of operation were lower than those before anesthesia induction, Da-jvO_2_ was higher than those before anesthesia induction (*P* < 0.001), the state entropy, reaction entropy, and CERO_2_ at the end of operation were higher than those at the end of operation, and Da-jvO_2_ was lower than those at the end of operation (*P* < 0.001). See Table 1.

### 3.2. Incidence of Postoperative Hyperalgesia in Different Patients

Postoperative hyperalgesia occurred in 40 of 266 patients; the incidence rate was 15.04% (40/266). Long-term sleep disturbance before operation, operation time, remifentanil dosage, 30 min during operation, state entropy at the end of operation, reaction entropy, CERO_2_, and Da-jvO_2_ are related to postoperative hyperalgesia (*P* < 0.05). See Table 2.

### 3.3. Multivariate Analysis of Postoperative Hyperalgesia

The items with statistically significant difference in 2.2 were tested for multicollinearity. It was found that there was multicollinearity between the intraoperative 30 min state entropy, reaction entropy, CERO_2_, Da-jvO_2_, and the value Vif at the end of the operation > 5. There was multicollinearity between the state entropy and reaction entropy at the end of the operation. There was multicollinearity between CERO_2_ and reaction entropy at the end of the operation. The intraoperative 30 min state entropy, reaction entropy CERO_2_, Da-jvO_2_, and state entropy and reaction entropy at the end of operation. Finally, the long-term sleep disorder before operation, the amount of remifentanil after operation, the reaction entropy at the end of operation, and CERO_2_ were corrected into the logistic model. See Tables 3 and 4.

RETRACTED

### 3.4. Establishment and Evaluation of Logistic Regression Model of Postoperative Hyperalgesia

(1) The establishment of (1) logistic regression model: logit(*P*) = −25.461 + 0.942 × remifentanil dosage + 1.292 × reaction entropy at the end of operation + 1.350 × CERO_2_ at the end of operation. (2) The total validity of logistic regression model: the likelihood chi-square ratio = 302.341, DF = 7, *P* < 0.001, the model is effective. The results of Wald test showed that Wald *χ*^2^ = 321.07, DF = 4, *P* < 0.001, and the coefficient difference of regression equation was statistically significant. (3) Goodness-of-fit test of (3) logistic regression equation: the goodness-of-fit test of Hosmer-Lemeshow shows that *χ*^2^ = 6.327, DF = 8, *P* = 0.628, which indicates that the model has a good degree of fit. See Table 5

### 3.5. Predictive Value of Reaction Entropy and CERO_2_ at the End of Operation for Postoperative Hyperalgesia

The data of patients with hyperalgesia were taken as positive data, and the data of patients without hyperalgesia were taken as negative data. ROC analysis showed that the AUC value of postoperative hyperalgesia predicted by reaction entropy and CERO_2_ at the end of operation was 0.851, which was greater than the reaction entropy at the end of operation (*χ*^2^ = 3.847, *P* = 0.036) and CERO_2_ (*χ*^2^ = 2.589, *P* = 0.010). See Figure 1 and Table 6.

## 4. Discussion

The causes of remifentanil induced hyperalgesia are related to high dose, long anesthesia time, and sudden change of concentration. At present, its mechanism has not been clarified [9]. Related studies have found that remifentanil can activate protein kinase C and calcium/calmodulin-dependent protein kinase II, promote the phosphorylation of N-methyl-D-aspartate receptor (NMDAR) subunit, increase the content of excitatory neurotransmitter glutamate, regulate the level of primary dynorphin mRNA at the spinal cord level, activate bradykinin receptor in the spinal cord, increase the hypersensitivity of the body to pain, and induce hyperalgesia [10]. However, there is no clinical report on how to predict remifentanil-induced hyperalgesia. In order to further prevent remifentanil-induced hyperalgesia, this study attempts to predict by monitoring relevant indicators during anesthesia. Studies have shown that controlling BIS target value at 50~59 under total intravenous anesthesia, compared with controlling BIS target value at 40~49, can effectively alleviate hyperalgesia of patients undergoing lower abdominal laparotomy [11]. Therefore, it is speculated that insufficient anesthesia depth will affect postoperative hyperalgesia. However, which objective index can be used to monitor the anesthesia depth of patients to assess the risk of hyperalgesia is still inconclusive clinically. Entropy index is a new type of EEG monitoring index. Collecting EEG and frontal EMG signals of different frequencies forms state entropy and reaction entropy, which can reflect the complexity and irregularity of the body system [12]. The state entropy is calculated according to EEG, and the reaction entropy is a comprehensive index of EEG and frontalis electromyography, which can better reflect the depth of anesthesia. The monitoring results of this study show that the state entropy and reaction entropy at 30 min during operation and at the end of operation are lower than those before anesthesia induction, but higher than 30 minutes during the operation, which is similar to the research results of Xu et al. [13] and Zhou et al. [14]. In addition, this study also found that the state entropy and reaction entropy at the end of operation were related to postoperative hyperalgesia (*P* < 0.05), which confirmed the above speculation. The main reason may be that when the depth of anesthesia is insufficient, the body is prone to the stress reaction of operation injury, especially when the operation time is longer (the operation time is ≥2 h), and this stress reaction is more obvious, which can disturb the normal pain mechanism of the body and is difficult to recover [15], and the electrical signal conduction in the central nervous system is one of the key links to regulate the pain response. When remifentanil activates NMDAR in the postsynaptic membrane, it can cause a large influx of Ca2+. It is reabsorbed by mitochondria to generate superoxide ions to activate calcium-dependent protein kinases; at the same time, related kinases can regulate NMDAR phosphorylation and then control the current signal of the central nervous system, showing the increase or decrease of state entropy and reaction entropy [16]. However, some studies have pointed out that postoperative hyperalgesia caused by remifentanil anesthesia maintenance is related to many factors such as operation time [17]. This study also found that, after correcting the long-term sleep disorder before operation and the operation time, the reaction entropy at the end of operation still entered the equation, which objectively indicated that the entropy index might provide reference for clinical evaluation of postoperative hyperalgesia risk.

RETRACTED

In addition, it has been clinically confirmed that the central nervous system can bidirectionally regulate and control external noxious stimuli through the downward inhibition and facilitation system. If noxious stimuli persist, it can trigger downward inhibition and facilitation and promote a new balance between the spinal cord and downward modulation effect, that is, hyperalgesia [18]. The changes of cerebral oxygen metabolism caused by operation and application of remifentanil can directly affect the regulatory function of the central nervous system [19]. Therefore, monitoring the cerebral oxygen metabolism during remifentanil anesthesia maintenance may provide reference for clinical assessment of hyperalgesia risk. Da-jvO_2_ and CERO_2_ are important indexes reflecting cerebral blood flow and cerebral oxygen consumption, which are often used to evaluate cerebral oxygen metabolism in general anesthesia. The research showed that Da-jvO_2_ increased and CERO_2_ decreased after anesthesia, suggesting that the metabolic level and oxygen consumption of brain tissue decreased and gradually recovered to the preoperative state with the end of the operation [20]. The results showed that Da-jvO_2_ was higher than that before anesthesia induction and CERO_2_ was lower than that before anesthesia induction at 30 min during operation, while Da-jvO_2_ and CERO_2_ gradually recovered at the end of operation, which was consistent with the above research results. This study also found that Da-jvO_2_ levels were generally lower and CERO_2_ levels were generally higher in patients with hyperalgesia at 30 minutes during operation and at the end of operation. This may be due to the need to choose the appropriate anesthesia depth during remifentanil anesthesia maintenance. On the one hand, sedation is used to suppress nociceptive stimulus afferent and stress response activation [21]; on the other hand, brain oxygen metabolism is reduced to improve central nervous system hypoxia tolerance. If brain oxygen metabolism is not effectively reduced during operation and brain oxygen metabolism recovers too quickly after anesthesia drugs are stopped, it may affect central nervous system function due to insufficient blood oxygen supply, which eventually leads to downward inhibition and facilitation, resulting in postoperative hyperalgesia [22]. In this study, the multivariate logistic regression model analysis showed that the risk of postoperative hyperalgesia increased with the increase of reaction entropy and CERO_2_ at the end of operation. Continuing the ROC analysis, the AUC value of the combined prediction of reaction entropy and CERO_2_ at the end of operation was 0.851, which was higher than that predicted by a single index (*P* < 0.001), indicating that entropy index and cerebral oxygen metabolism had high predictive value for postoperative hyperalgesia maintained by remifentanil anesthesia. However, postoperative hyperalgesia is related to many factors such as individual differences of patients. Long-term sleep disturbance before operation, operation time, 30 min state entropy, response entropy, CERO_2_, Da-jvO_2_, and state entropy and Da-jvO_2_ at the end of the operation are correlated. But this correlation is an uncertain relationship. There may be more complex relationships between observations. Although some confounding factors have been corrected in this study, the objectivity of the conclusion still needs to be demonstrated.

RETRACTED

To sum up, entropy index and cerebral oxygen metabolism are independently related to postoperative hyperalgesia, and joint monitoring can provide reference for clinical evaluation of postoperative hyperalgesia risk. When the reaction entropy is greater than 54.23, CERO_2_ is greater than 34.14%, or the total amount of remifentanil is ≥30 *μ*g/kg at the end of the operation, we should be highly alert to the occurrence of postoperative hyperalgesia and strengthen the management of postoperative analgesia.

## Figures and Tables

**Figure 1:** ROC analysis.

**Table 1:** Comparison of entropy index and cerebral oxygen metabolism before and after anesthesia ($\bar{x}\pm s$).

Time	Entropy index		Cerebral oxygen metabolism	
	State entropy	Reaction entropy	Da-jvO_2_ (ml/l)	CERO_2_ (%)
Before induction of anesthesia	90.18 ± 1.76	93.01 ± 1.83	43.40 ± 6.84	40.01 ± 4.17
30 min during operation	47.69 ± 5.03^a^	50.12 ± 5.19^a^	55.57 ± 7.94^a^	30.13 ± 4.18^a^
At the end of the operation	49.12 ± 5.21^ab^	52.04 ± 5.46^ab^	52.08 ± 7.06^ab^	32.82 ± 3.63^ab^
*F*	8365.011	7794.024	196.203	428.659
*P*	<0.001	<0.001	<0.001	<0.001

Note: compared with before anesthesia induction, ^a^*P* < 0.05; compared with 30 min during operation, ^b^*P* < 0.05.

**Table 2:** The incidence of postoperative hyperalgesia in different patients was *n* (%).

Factor	Example number (*n* = 266)	Hyperalgesia (*n* = 40)	*χ* ^2^	*P*
Age (years)				
<16	12	3 (25.00)	4.790	0.091
16~60	179	21 (11.73)		
>60	75	16 (21.33)		
Sexuality				
Man	146	21 (14.38)	0.108	0.742
Woman	120	19 (15.83)		
Body mass index (kg/m^2^)				
<24	104	17 (16.35)	0.229	0.632
≥24	162	23 (14.20)		
Degree of education				
Junior high school and below	101	15 (14.85)	0.006	0.997
High school or technical secondary school	93	14 (15.05)		
College degree or above	72	11 (15.28)		
A history of smoking				
Yes	47	9 (19.15)	0.755	0.385
No	219	31 (14.16)		
History of alcohol abuse				
Yes	25	4 (16.00)	0.023	0.879
No	241	36 (14.94)		
Long sleep disturbance before surgery				
Yes	158	30 (18.98)	4.752	0.029
No	108	10 (9.26)		
The way of anesthesia maintenance				
Thoracic cannula for general anesthesia	128	20 (15.63)	0.196	0.907
Static composite anesthesia	32	4 (12.50)		
All by intravenous anesthesia	106	16 (15.09)		
ASA classification				
I level	129	18 (13.95)	0.404	0.817
II level	116	18 (15.52)		
III level	21	4 (19.05)		
Operation time (h)				
<2	198	24 (12.12)	5.156	0.023
≥2	68	16 (23.53)		
Operative site				
Body surface	142	22 (15.49)	0.119	0.989
Arms and legs	55	8 (14.55)		
Body cavity	44	6 (13.64)		
Other	25	4 (16.00)		
The dosage of remifentanil (*μ*g/kg)				
<30	181	21 (11.60)	5.232	0.022
≥30	85	19 (22.35)		
State entropy				
Low levels before the induction of anesthesia	130	18 (13.85)	0.283	0.595
High levels before the induction of anesthesia	136	22 (16.18)		
Low intraoperative level of 30 min	128	12 (9.38)	6.192	0.013
High intraoperative level of 30 min	138	28 (20.29)		
Low levels at the end of the surgery	135	14 (10.37)	4.674	0.031
High level at the end of the surgery	131	26 (19.85)		
Reaction entropy				
Low levels before the induction of anesthesia	132	17 (12.88)	0.956	0.328
High levels before the induction of anesthesia	134	23 (17.16)		
Low intraoperative level of 30 min	133	14 (10.53)	4.237	0.040
High intraoperative level of 30 min	133	26 (19.55)		
Low levels at the end of the surgery	135	13 (9.63)	6.275	0.012
High level at the end of the surgery	131	27 (20.61)		
Da-jvO_2_ (ml/l)				
Low levels before the induction of anesthesia	134	18 (13.43)	0.544	0.461
High levels before the induction of anesthesia	132	22 (16.67)		
Low intraoperative level of 30 min	130	27 (20.77)	6.538	0.011
High intraoperative level of 30 min	136	13 (9.56)		
Low levels at the end of the surgery	133	29 (21.80)	9.534	0.002
High level at the end of the surgery	133	11 (8.27)		
CERO_2_ (%)				
Low levels before the induction of anesthesia	131	18 (13.74)	0.340	0.560
High levels before the induction of anesthesia	135	22 (16.30)		
Low intraoperative level of 30 min	129	11 (8.53)	8.309	0.004
High intraoperative level of 30 min	137	29 (21.17)		
Low levels at the end of the surgery	134	14 (10.45)	4.453	0.035
High level at the end of the surgery	132	26 (19.70)		

Note: state entropy, reaction entropy, Da-jvO_2_, and CERO_2_ are bounded by the mean value, ≤mean value is low level, >mean value is high level; “-” means that there is at least one lattice theoretical number *T* ≤ 1, and there is no *χ*^2^ value.

RETRACTED

**Table 3:** Assignment.

Variable		Assignment
Dependent variable	Postoperative hyperalgesia	No = 0, yes = 1
Independent variable	The long-term sleep disorder before operation	No = 0, yes = 1
	Operation time	Actual value
	The dosage of remifentanil	Actual value
	Response entropy at the end of the surgery	Actual value
	CERO_2_ at the end of the surgery	Actual value

**Table 4:** Multivariate analysis of postoperative hyperalgesia.

Factor	*β*	S.E.	Wald *χ*^2^	*P*	OR	95% CI
Long sleep disturbance before surgery	0.472	0.392	1.450	0.618	1.603	0.428~6.005
Operation time	0.588	0.411	2.048	0.326	1.801	0.576~5.629
The dosage of remifentanil	0.942	0.325	8.408	0.003	2.566	1.369~4.810
Response entropy at the end of the surgery	1.292	0.372	12.065	<0.001	3.641	2.003~6.617
CERO_2_ at the end of the surgery	1.350	0.398	11.500	<0.001	3.856	1.858~8.003
Constant term	-25.461					

**Table 5:** Table of randomness of the Hosmer-Lemeshow test.

Test times	Postoperative hyperalgesia = yes		Postoperative hyperalgesia = no		Total number of cases
	Actual observation value	Model expectation value	Actual observation value	Model expectation value	
1	26	25.34	14	14.66	40
2	21	21.06	31	30.94	52
3	20	20.31	16	15.69	36
4	16	15.64	25	25.36	41
5	28	27.36	19	19.64	47
6	13	12.45	22	22.55	35
7	22	20.98	24	25.02	46
8	23	22.76	16	16.24	39
9	15	15.69	30	29.31	45
10	19	18.37	23	23.63	42

**Table 6:** Predictive value of reaction entropy and CERO_2_ at the end of operation for postoperative hyperalgesia.

Parameter	AUC value	95% CI	*χ* ^2^	*P*	Cutoff value	Sensitivity (%)	Specificity (%)
Reaction entropy	0.778	0.724~0.844	7.344	<0.001	>54.23	77.50	74.78
CERO_2_	0.724	0.666~0.777	5.258	<0.001	>34.14%	62.50	77.43
Unite	0.851	0.802~0.891	8.098	<0.001		80.00	80.53

## Data Availability

The labeled dataset used to support the findings of this study is available from the corresponding author upon request.
